# Artificial Intelligence Limb Rehabilitation System on Account of Virtual Reality Technology on Long-Term Health Management of Stroke Patients in the Context of the Internet

**DOI:** 10.1155/2022/2688003

**Published:** 2022-05-23

**Authors:** Yu Bai, Fang Liu, Hua Zhang

**Affiliations:** ^1^Department of Neurology, Changzhou No.2 People's Hospital, Changzhou, 213000 Jiangsu, China; ^2^Department of Neurosurgery, Changzhou No.2 People's Hospital, Changzhou, 213000 Jiangsu, China

## Abstract

This study was aimed at discussing artificial intelligence (AI) limb rehabilitation system on account of virtual reality (VR) on long-term health management of stroke patients. In the study, AI limb rehabilitation system on account of VR technology was compared with traditional drug therapy, and effects of the two therapies on long-term health management of stroke patients were compared. Fifty patients with stroke in the hospital were randomly divided into experimental group and control group with 25 patients in each group. Patients in experimental group were treated with AI limb rehabilitation system on account of VR technology, and those in control group were treated with traditional drug therapy. To compare and judge the recovery of patients' physical ability, patients in the two groups were compared in physical movement ability and daily living activity ability after 10-week treatment. After 10-week treatment, Fugl-Meyer assessment-upper extremity (FMA-UE), Fugl-Meyer assessment-lower extremity (FMA-LE), the Hong Kong version of functional test for the hemiplegic upper extremity (FTHUE-HK), Barthel index (BI) daily living (ADL) activities, and Berg balance scale (BBS) in control group were lower than those in experimental group, but the score of MWS was higher than that of experimental group (*P* < 0.05). AI limb rehabilitation system on account of VR technology could effectively recover the daily health management of stroke patients, and its effect was significantly higher than that of traditional drug therapy. This method could be popularized in clinic.

## 1. Introduction

Cerebral stroke is commonly known as stroke in traditional Chinese medicine. Several factors contribute to a cerebral stroke to certain areas of brain tissue, which cause damage to brain tissue [1]. Stroke can be divided into cerebral ischemic stroke and cerebral hemorrhage according to different symptoms. The incidence of cerebral ischemic stroke was much higher than that of cerebral hemorrhage, which accounts for about 70% of all strokes [2, 3]. Stroke was an emergency and may cause death within days or even hours after onset. Some patients still suffer from relapse after treatment, which requires long-term follow-up management [4, 5].

For patients, stroke is prone to cause disability or apoplexy sequelae [6]. The symptoms mainly include hemiplegia, paralysis, and loss of speech function, self-care ability, and mobility [7]. Patients with mild symptoms can fully recover their normal working and living ability after early corresponding rehabilitation treatments [8]. At present, the main means of exercise rehabilitation therapy were drug therapy and exercise rehabilitation, which mainly rely on patients, their families, and nursing staff to carry out self-discipline and supervision management [9]. With the development of artificial intelligence (AI) technology and the gradual improvement of virtual reality (VR) technology, there are mature virtual interactive products that can provide more immersive interactive and personalized scenes according to users' conception at present. They can make up for the boring, repetitive, and insufficient feedback and insufficient task orientation of traditional rehabilitation training [10–12].

Under the logistics network environment, sensor technology was widely used, which makes the VR technology have further development space in the field of remote control. Current VR technology can provide users with all kinds of training or other types of fun scenarios on account of designs that are closer to real life according to designers, some personalized training time tasks, or personalized learning modes. These learning and training modes that cannot be provided by traditional treatment schemes can provide a novel and interesting rehabilitation scheme for the prognosis of motor dysfunction in stroke patients. At present, the actual effect of VR technology in the long-term health management of stroke patients is not clear.

In this study, 50 patients with stroke in the hospital were randomly divided into experimental group and control group. This study innovatively puts forward the artificial intelligence limb rehabilitation system based on virtual reality to train the experimental group, aiming at exploring its advantages in health management of stroke patients.

## 2. Materials and Methods

### 2.1. Research Objects

In this study, 50 patients with stroke from May 2019 to December 2020 were selected as research objects. In experimental group, there were 18 males and 7 females, aged 47~68 years old, with an average age of 54.2 ± 13.7 years old and an average onset time of 141.54 ± 38.28 days. There were 21 patients with cerebral infarction, 4 patients with cerebral hemorrhage, 14 patients with upper extremity (UE) hemiplegia, and 11 patients with lower extremity (LE) hemiplegia. In the control group, there were 25 patients with 15 males and 10 females, aged 43~67 years old, with an average age of 56.9 ± 14.6 years old and an average onset time of 132.29 ± 41.62 days. There were 23 patients with UE hemiplegia, 2 patients with cerebral hemorrhage, 13 patients with UE hemiplegia, and 12 patients with LE hemiplegia. This study had been approved by ethics committee of hospital, and patients' families were informed of it and signed informed consents.

Inclusion criteria were as follows: First, the symptom of patients was in line with *Key Points of Diagnosis of Various Cerebrovascular Diseases* in the 4th National Academic Conference on Cerebrovascular Diseases in 1996, and it was confirmed by brain computed tomography or nuclear magnetic resonance examination [13]. Second, all patients had primary stroke. Third, patients had UE and LE hemiplegia. Fourth, patients were clearly conscious and could fully understand test requirements and effectively cooperate. Fifth, patients voluntarily participated in the study and signed informed consents.

Exclusion criteria were as follows: First, patients had serious cardiovascular diseases. Second, patients were not suitable for exercise such as lower limb fracture or surgery. Third, patients had severe cognitive dysfunction and deep sensory impairment. Fourth, patients had myocardial infarction, heart failure, and other diseases recently. Fifth, patients had unstable vital signs and organ failure. Sixth, patients could not stay in the hospital all the time and complete the 10-week rehabilitation program.

### 2.2. Rehabilitation Therapy

In the control group, patients received general traditional rehabilitation training methods, and professional medical staff customized personalized rehabilitation training plans according to specific conditions of patients. Specific projects of rehabilitation training were traditional medicine, physical therapy, speech therapy, and occupational therapy (OT). These four specific projects were the traditional treatments for the prognosis of stroke patients. OT, as a kind of training task, mainly provided patients with necessary training tasks through selective operation activities, so as to meet the recovery of various physiological functions. The followings were its main training programs: upper limb fetching exercises, arms forward, and back rotation exercises for shoulder and elbow joints; screwing screws, grabbing objects, and others for finger flexibility; steering training, motion maintenance training, standing balance training, sitting up training, and bridge movement for lower limb joint; and roller training, dressing training, routine living equipment training, and routine walking training which includes walking up and down stairs, lateral walking, cross walking, and others for daily life [14].

In the experimental group, patients received training tasks on account of VR technology in addition to traditional treatments for stroke patients such as traditional medicine, physical therapy, speech therapy, and OT. VR system was divided into motion sensor, motion capture suit, computer monitor, VR digital training system, and training evaluation software. Medical staff wore motion capture suits according to patients' training and physical conditions during general training and fixed motion sensors at the corresponding joints of the body. Motion capture was then performed according to patients' real-time exercise rehabilitation training, transferred to computers through three dimensional (3D) spatial parameters, motion changes, and virtual motion system, and fed back to monitors.

At present, VR digital training system mainly consists of multitouch training table and universal treadmill. Multitouch training table is mainly for upper limb training of patients. It has a large number of training modules, including fruit cutting games, driving games, whac-a-mole games, picture combination games, goal tracking games, and coordination training. As the main equipment for limb training, universal treadmill is collected and fed back the walking and running data of patients during rehabilitation training. It can be matched with maze games, balance training, running training, obstacle avoidance, and so on. At the same time, this kind of training module supports the modification of training time and difficulty and combines with the training evaluation software, and the training content can be personalized and adjusted according to the training effect of patients. A training experience integrating interest, creativity, immersion, and interactivity can be created by providing patients with auditory, tactile, and visual sensory stimulation. In this way, patients can be actively immersed in the training content and maximize the training effect. VR training lasts 40~60 min a day, 5 days a week for 10 weeks.

### 2.3. Observation and Evaluation of Curative Effect

The exercise ability of patients in two groups was evaluated prior and post 10-week rehabilitation treatment. Fugl-Meyer assessment-upper extremity (FMA-UE), Fugl-Meyer assessment-lower extremity (FMA-LE), the Hong Kong version of functional test for the hemiplegic upper extremity (FTHUE-HK), Barthel index (BI) of activities of daily living (ADL), Berg balance scale (BBS), and 10 m maximum walking speed (MWS) were used in this study. FMA-UE and FMA-LE belonged to FMA. The mobility of the upper and lower limbs could be assessed by them separately. It could be selected according to hemiplegia patients. The lower the score was, the more severe the injury degree of upper and lower limbs would be. The upper limb function test of hemiplegia mainly aimed at the evaluation of the functional recovery ability of Chinese patients with stroke or hemiplegia in the upper limb rehabilitation training. It had high pertinence and credibility. Patients' upper limb mobility could be graded according to 12 items, and the higher the grade was, the better the upper limb mobility would be. BI scored patients' ADL through a series of independent behavioral evaluations. The program was divided into 10 items which included eating, washing, dressing, going to the toilet, dressing, walking, defecating, urinating, moving utensils, and walking up and down stairs. The higher the score was, the stronger the independent living ability would be. BBS evaluated patients' lower limb balance ability through 14 evaluation criteria. The higher the score of patients was, the better their behavioral ability would be. 10 m MWS mainly aimed at the evaluation of patients' lower limb mobility. It selected a barrier-free route with a straight line distance of 16 m and calibrated it at the starting point, 3 m, 13 m, and the end point. It recorded the time required 3 m~13 m by selecting a barrier-free route with a straight line distance of 16 m. This process was repeated 3 times. Appropriate rest could be carried out in the middle, and the shortest time was selected as the final time [15–18].

### 2.4. Statistical Methods

Statistical product and service solutions 19.0 version was used for data analyses, measurement data were expressed by $\bar{\text{x}}\pm \text{s}$, counting data were expressed by %, and pairwise comparison adopted 1 factor variance analyses. *P* < 0.05 indicated significant differences.

## 3. Results

### 3.1. Comparison of Evaluation Scale Results

The comparison results of specific clinical data statistics of patients were shown in Figure 1. There were no significant differences in individual clinical data between the two groups (*P* > 0.05), which indicated comparability.

### 3.2. Score Comparison of Experimental Results

The evaluation tables of prior and post rehabilitation treatment of all patients in two groups were compared, and the specific results were shown in Figures 2–7.

In Figure 2, the scores of prior and post treatment of control group were 34.77 ± 0.58 and 41.82 ± 0.79, respectively, and those of experimental group were 35.26 ± 0.57 and 47.46 ± 0.48, respectively. The data of two groups were compared, and results showed significant statistical differences (*P* < 0.05).

In Figure 3, in the lower limb motor function evaluation scale, the scores of prior and post treatment of control group were 18.36 ± 1.33 and 27.53 ± 1.69, respectively, and those of experimental group were 18.20 ± 1.62 and 32.63 ± 1.36, respectively. There were significant statistical differences between the two groups (*P* < 0.05).

In Figure 4, in the score of hemiplegic upper limb function test (Hong Kong version), prior and post treatment in control group were 3.72 ± 0.48 and 4.06 ± 0.52, respectively, and those of experimental group were 3.27 ± 0.51 and 4.84 ± 0.56, respectively. The results showed significant statistical differences (*P* < 0.05).

In Figure 5, for BI, the scores of prior and post treatment of control group were 65.98 ± 1.38 and 72.51 ± 1.52, respectively, and those of experimental group were 64.48 ± 1.57 and 78.32 ± 1.32, respectively. There were significant statistical differences between the two groups (*P* < 0.05).

In Figure 6, BBS showed that the scores prior and post treatment of control group were 23.75 ± 1.86 and 34.36 ± 1.63, respectively, and those of experimental group were 24.47 ± 1.58 and 41.58 ± 1.56, respectively. The results of data comparison between the two groups showed significant statistical differences (*P* < 0.05).

In Figure 7, in 10 m MWS, the scores of prior and post treatment of control group were 77.43 ± 4.81 and 60.27 ± 3.95, respectively, and those of experimental group were 79.03 ± 5.72 and 56.51 ± 4.26, respectively. The results showed significant statistical differences between the two groups (*P* < 0.05).

According to the above results, AI limb rehabilitation system on account of VR technology had a better therapeutic effect on the prognosis rehabilitation training of stroke patients compared with the traditional rehabilitation training.

## 4. Discussion

The behavioral rehabilitation of patients with cerebral apoplexy had always been one of the important problems for patients and their families. After stroke, a large number of patients had hemiplegia, paralysis, loss of self-care ability, and other sequelae. They seriously affect daily lives and bring a lot of inconvenience to themselves and their families. Therefore, it was very important to establish a set of scientific and effective motor rehabilitation management for stroke patients. Therefore, this study intended to build a rehabilitation training system that could not only meet the needs of daily rehabilitation training but also improve patients' training initiative and dependence. In recent years, with the hot and development of VR technology, it was possible to construct 3D space and supporting interactive environment without being affected by environmental factors, which was basically consistent with the requirements of this study. Therefore, AI limb rehabilitation system on account of VR technology in the rehabilitation training of stroke patients was one of the future development trends [19].

The objective of this study was to compare AI limb rehabilitation system on account of VR technology with traditional drug therapy on the rehabilitation of limb movement ability of stroke patients. 50 patients were randomly divided into control group and experimental group and underwent rehabilitation training for 10 weeks, respectively. Compared with traditional treatment, AI limb rehabilitation system on account of VR technology could better improve the rehabilitation efficiency of stroke patients and play an obvious role in the recovery of all physiological motor functions of patients. The reasons could be the followings: first, AR limb rehabilitation technology on account of VR technology could track and analyze the rehabilitation training activities of patients in time, adjust the exercise mode and difficulty in time, take into account the individual needs of users, and avoid a lot of homogeneous meaningless or low-intensity training. Second, it could bring more fun, guarantee a certain novelty, improve the dependability of the rehabilitation training in patients with cerebral apoplexy and initiative, and thus improve the effect of rehabilitation training brought about by the unique immersive VR technology and creativity to users' touch, vision, and hearing stimulated at the same time. Third, it could correct users' trained actions in time with the help of AI in computer systems. It had higher patience and carefulness compared with traditional rehabilitation training, could ease users' mood through sound effects and environment transformation at the same time, and avoid the psychological anxiety caused by a long time training. Fourth, it was easy to operate and could adopt different operating systems according to the users' different modules. At the same time, it was not limited to the requirements of the sites and could move thousands of miles between the square inch through VR technology. Users could not only play the rehabilitation training but also train work and life abilities after rehabilitation by various scenes through the establishment of the corresponding positive feedback mechanism of the system. However, there were also many problems in it: first, the price was too expensive; second, device security should be considered; and third, there were fewer development modules. At present, VR technology was an emerging industry and its supporting software is not perfect, so it still needs further development and improvement in clinical use.

Faria et al. [20] designed a set of virtual city on account of VR technology for the training of Addenbrooke's cognitive ability of stroke patients. The results demonstrated that VR improved patients' overall cognition, attention, and executive performance more significantly than traditional drug therapy. Lin et al. [21] conducted a randomized controlled trial on the influence of upper and lower limb muscles and emotions in early rehabilitation of stroke patients by using VR technology. VR technology had a stronger effect on emotional state and muscle strength in early rehabilitation training of stroke patients.

## 5. Conclusion

This study was aimed at discussing AR limb rehabilitation system on account of VR technology in the prognosis of stroke patients. The clinical value of it was judged by comparing the rehabilitation effect of the rehabilitation system with that of ordinary stroke patients. The system had a better effect on the prognosis of stroke patients than ordinary training and had a high clinical value. The deficiency of this paper was that the artificial intelligence limb rehabilitation system based on virtual reality technology is expensive and not suitable for large-scale clinical popularization. On the other hand, because the system was a new industry, the types of matching software are not perfect at present. Therefore, although the experiment proves that this method has a high rehabilitation effect, it was still recommended to wait for the development of virtual reality technology. This study provided a new direction for the prognosis and rehabilitation of patients with cerebral apoplexy, the corresponding experimental data, and some clinical experience for the development of technology and clinical use in the future.

## Figures and Tables

**Figure 1:** Comparison of clinical data of patients. (a) showed the comparison of stroke types; (b) showed the comparison of hemiplegia types; (c) showed the comparison of average age of patients; (d) showed the comparison of sex of patients; and (e) showed the comparison of the mean onset time of patients. Compared with control group, experimental group showed *P* > 0.05.

**Figure 2:** Comparison of results of FMA-UE. ^∗^Compared with control group, *P* < 0.05.

**Figure 3:** Comparison of results of FMA-LE. ^∗^Compared with control group, *P* < 0.05.

**Figure 4:** Comparison of results of FTHUE-HK. ^∗^Compared with control group, *P* < 0.05.

**Figure 5:** Comparison of BI results. ^∗^Compared with control group, *P* < 0.05.

**Figure 6:** Comparison of BBS. ^∗^Compared with control group, *P* < 0.05.

**Figure 7:** Comparison of 10 m MWS. ^∗^Compared with control group, *P* < 0.05.

## Data Availability

The data used to support the findings of this study are available from the corresponding author upon request.
